The article "Ultrasonic Imaging of Carotid Inflammatory Plaque with Superparamagnetic Nanoparticles" was retracted in 2023. Reasons: unreliable results or conclusions; concerns about the data; concerns about the peer review; concerns about the citations.

# Ultrasonic Imaging of Carotid Inflammatory Plaque with Superparamagnetic Nanoparticles

**DOI:** 10.1155/2021/9685660

**Published:** 2021-12-02

**Authors:** Wei Li, Jiang Wu, Mingjin Guo, Jing Shang

**Affiliations:** ^1^Department of Vascular Surgery, The Affiliated Hospital of Qingdao University, Qingdao City 266000, China; ^2^Department of Health Management, The Affiliated Hospital of Qingdao University, Qingdao City 266000, China

## Abstract

Chronic inflammation can stimulate the formation and progression of atherosclerotic plaques and increase the vulnerability of plaques. However, there are few studies on the changes of carotid inflammatory plaques during treatment. Our study attempted to investigate the use of superparamagnetic iron oxide nanoparticle (SPION) ultrasound imaging to detect the expression of vascular cell adhesion molecule-1 (VCAM-1) in patients with carotid plaques and analyze the effects of SPION ultrasound imaging in inflammatory plaque visualization effect. SPION microbubble contrast agents have good imaging effects both in vivo and in vitro. We conjugated the VCAM-1 protein to the microbubbles wrapped in SPIONs to form SPIONs carrying VCAM-1 antibodies. Observe the signal intensity of SPIONs carrying VCAM-1 antibody to arteritis plaque. The results showed that the SPION contrast agent carrying VCAM-1 antibody had higher peak gray-scale video intensity than the other two groups of contrast agents not carrying VCAM-1 antibody. It shows that SPIONs have excellent imaging effects in ultrasound imaging, can evaluate the inflammatory response of arterial plaque lesions, and are of great significance for the study of carotid inflammatory plaque changes.

## 1. Introduction

Carotid artery plaque (CAP) is the deposition of fat and calcium on the inner wall of the carotid artery, which is an important manifestation of carotid atherosclerosis. The rupture of atherosclerotic plaque can lead to thrombosis and cause cardiovascular and cerebrovascular events [1]. Hyperlipidemia is closely related to CAP disease. Inflammation can lead to plaque formation and accelerate the rate of plaque formation [2]. Therefore, the identification of inflammatory plaques before the occurrence of cardiovascular and cerebrovascular events plays an important role in the prevention and diagnosis of cardiovascular and cerebrovascular diseases.

Clinical imaging techniques for atherosclerotic plaque examination mainly include digital subtraction angiography (DSA), intravascular ultrasound imaging (IUI), magnetic resonance angiography (MRA), color Doppler ultrasound vascular examination (CDF), and computed tomography angiography (CTA) [3–5]. DSA is the “gold standard” for detecting CAP, but DSA is an invasive examination and of high cost and has complications. It can only judge the degree of stenosis of the arterial vessel lumen and cannot show the composition of the arterial vessel wall and atherosclerotic plaque. CTA and MRA can also determine the degree of carotid artery stenosis and can also evaluate vulnerable plaques, but due to the complicated inspection process and high cost, they have not been widely used in clinical practice. The advantages of ultrasound imaging are real-time, no trauma, no radioactivity, etc. It is currently the first choice for imaging diagnosis.

Although traditional ultrasound contrast agents are not poor in diagnostic accuracy, it is difficult to meet the requirements for accuracy, targeting, and specificity at the same time [6]. With the continuous development of ultrasound contrast agents, ultrasound imaging has made great progress in tissue perfusion of internal organs, tumor diagnosis, and inflammation detection. However, due to its low spatial resolution, the performance in the imaging results is not perfect [7]. Therefore, seeking the contrast agent with the best imaging effect is of great significance for the accurate detection of carotid plaque.

Magnetic nanoparticles are a new type of tracer material used in imaging diagnosis in recent years. When the surface of magnetic nanoparticles is modified by specific organic/inorganic polymers, their functions are more differentiated. For example, surface-modified particles can track some biologically active molecules that can specifically bind to the particle surface [8]. When a magnetic material is under the action of an external magnetic field, the originally oriented magnetic moment will be oriented, thus exhibiting paramagnetism [9]. Superparamagnetism means that its paramagnetic susceptibility is much higher than that of general paramagnetic materials under the action of an external magnetic field. Superparamagnetic iron oxide nanoparticles (SPIONs) are commonly used engineered biocompatible nanoparticles and have been approved by the FDA for use as contrast agents [10]. SPIONs can change the longitudinal and lateral relaxation time to increase image contrast and improve resolution [11]. SPIONs are mainly reported in magnetic resonance imaging, but rarely in ultrasound imaging. Therefore, this paper studies the imaging effect of SPIONs on carotid plaque ultrasound imaging.

## 2. Materials and Methods

### 2.1. Preparation of SPIONs

Nanometer Fe_3_O_4_ (Fe_3_O_4_) was synthesized by solvothermal reaction. Fe_3_O_4_·6H_2_O (1.089 g, 4.0 mmol), trisodium citrate (1.0 g, 3.4 mmol), and sodium acetate (2.4 g, 2.9 mmol) were added to a mixture of 45 mL of ethylene glycol and 15 mL of diethylene glycol. Stir rapidly at 22°C for 3 h. The resulting yellow solution was transferred to a 100 mL pressure cooker lined with polytetrafluoroethylene and heated at 200°C for 10 h. Then, cool naturally to 22°C. The obtained product was washed 3 times with ethanol and ultrapure water. Finally, the magnetic powder was dried in a vacuum oven at 60°C and then dispersed in water for further use. Disperse 1 mL of the magnetic particle solution evenly in 15 mL of water. Then, add 50 mL mercaptopropyltriethoxysilane and 150 mL ammonia (final concentration of 1.5%). Shake the mixture with a shaker at 2000 rpm for 1 minute. Store at 22°C for 18 hours. Use a magnet to collect the lower layer, and disperse it in 5 mL of water. Methoxypolyethylene glycol maleimide (5 mg) was mixed in the solution. After incubating for 5 hours, the suspension was separated, collected with a magnet, and washed 3 times to obtain PEGylated magnetic nanoparticles. The particle size is 50 nm, and the concentration is 0.1 mol/L.

### 2.2. Preparation of Microbubbles Wrapped in SPIONS

Polylactic acid (PLA, Mw = 10000) and polyvinyl alcohol (PVA, degree of polymerization = 1800, degree of alcoholysis = 89%) were purchased from Sigma-Aldrich. Dissolve 0.5 g PLA in 10 mL CHCl3. The SPION solution and the PLA solution were mixed uniformly, and then, 1 mL of double distilled water and 0.01 mL of span-80 were added to the PLA solution. The PLA solution was introduced into N2 (4 mL/min) at a constant rate, and during this process, ultrasonic cavitation was used for 2 min with a vibrometer (power 200 W/s) to obtain emulsion microbubbles. The emulsion microbubbles were poured into 50 mL of 5.0% PVA aqueous solution and stirred at 3000 r/min at 22°C for 2 h to obtain double emulsion microbubbles. After centrifugation at 1500 r/min at 20°C for 5 min, SPION microbubble contrast agent was obtained. As shown in Figure 1(a), the microbubbles encapsulate SPIONs, and Figure 1(b) is a partial enlarged photo of the microbubble membrane shells encapsulating SPIONs. SPIONs are evenly distributed in the polymer membrane shell.

### 2.3. SPION Carrying Antibodies to the Inflammatory Adhesion Molecule VCAM-1

SPION microbubbles were dispersed in double distilled water, which was put in a centrifuge at 1000 rpm for 3 minutes, and the supernatant was discarded. SPIONs were dispersed with 0.1 mol/L MES buffer (pH 6.0), which was placed in a centrifuge at 1000 rpm for 3 min, and the supernatant was discarded. SPIONs were dispersed again by 0.1 mol/L MES buffer (PH6.0). SPIONs were added with coupling agent EDC/NHS (PLGACOOH : EDC : NHS molar ratio 1 : 10 : 20) and incubated for 30 min. Rinse 2 times with MES buffer (pH 6.0), then rinse once with MES buffer (pH 8.0), centrifuge at 1000 rpm for 3 minutes, and discard the supernatant. The contrast agent was dispersed in MES buffer (pH 8.0) and added with excess anti-VCAM-1 antibody (Abcam, USA). The molar ratio of anti-VCAM-1 antibody : contrast agent was 50 : 1 and incubated for 2 h at room temperature. Rinse twice with PBS buffer to remove unbound anti-VCAM-1 antibody. Rinse twice with pH 7.0PBS buffer, centrifuge at 1000 rpm for 3 min, discard the supernatant to retain the lower layer, and add PBS to disperse.

### 2.4. In Vitro Contrast-Enhanced Ultrasound Imaging

In vitro experiments of SPION microbubbles were performed using self-made latex tubes. First, prepare degassed water, put the deionized water in an ultrasonic cleaner for 2 hours, and transfer the obtained degassed water to a water tank. A medical grade latex tube was placed below the surface of the degassed water. Next, the probe of the ultrasound imaging system was placed below the liquid surface and facing the latex tube. Use a syringe to suck up SPION microbubbles of different concentrations (1 × 10^2^, 1 × 10^4^, 1 × 10^6^, 1 × 10^8^, and 1 × 10^10^ particles/mL), and slowly inject them from one end of the latex tube. Compare the pulse sequence contrast mode to observe the longitudinal section of the latex tube. The control group was injected with saline.

### 2.5. Atherosclerosis Rat Model

Apolipoprotein E (ApoE) gene knockout rats were used to construct a rat model of atherosclerosis. We purchased 6-week-old male ApoE knockout rats from Zhishan (Beijing) Institute of Health Medicine. A total of 20 rats weighing 200-250 g were used to construct arteritis plaque rat model. All rats were housed in an SPF animal room at 22°C, where they can eat and drink freely. The light illumination-dark cycle was 12-12 h. D12492 high-fat feed was used for rat feed; the formula mainly contains 60% fat, 20% protein, and 20% carbohydrate. Daily regular feeding was given, and the feeding time was 16 weeks, respectively. In addition, 20 6-week-old male normal rats of the same weight were purchased as normal controls and fed an ordinary feed.

### 2.6. The Expression of VCAM-1 in Carotid Artery Was Examined by Contrast-Enhanced Ultrasound

The model rats were divided into groups A and B. Group A (10 rats) used SPIONs carrying VCAM-1 antibody to observe the results of carotid angiography, and group B (10 rats) used nontargeted SPIONs to observe the results of carotid angiography. After the contrast agent was injected into the rat, the images of each time period were recorded at 1 min, 5 min, 15 min, 30 min, 60 min, 2 h, 4 h, and 8 h. Origin8.0 software was used to draw the time-intensity curve.

### 2.7. Serum Lipid Determination

Blood was drawn from the tail vein before the experiment and 16 weeks after the experiment. The upper serum was taken to test the total cholesterol (TC) and low-density lipoprotein cholesterol (LDL-C) of the rats.

### 2.8. Pathological Examination

Rats were given inhaled isoflurane for induction anesthesia before general anesthesia. After the rats were quiet, the rats were anesthetized by intraperitoneal injection with 0.1 ml of 1% thiopentone injection (diluted with 0.9% normal saline and maintained anesthesia for about 20 minutes). After successful anesthesia, the rat was fixed on the dissection table. Routinely disinfect the rat's neck and spread towels. The neck skin of the rat was cut longitudinally to expose the carotid artery. After the carotid artery was completely peeled off, it was quickly fixed with 4% paraformaldehyde solution. After HE staining, the carotid artery plaque was observed and compared with the index of the ultrasound contrast result.

### 2.9. Statistical Analysis

SPSS23.0 software was used to analyze the data. Classified data were expressed as *n* (%), and the *χ*^2^ test was used. Quantitative data is represented by (*x* ± *s*), using a *t*-test. *P* < 0.05 is considered statistically significant.

## 3. Results and Discussion

### 3.1. Extracorporeal Ultrasound Imaging Effect

Different concentrations of SPION contrast agents were used to perform in vitro ultrasound imaging of the longitudinal section of the latex tube.  Figure 2(a) shows that compared with the control group, SPIONs have obvious punctate echoes in the latex lumen, and the echoes continue to increase as the concentration of the contrast agent increases (see Figure 2(b)). It is suggested that the SPION contrast agent has good imaging effect in vitro, so we will analyze the imaging effect of SPION contrast agent on rat carotid artery plaque.

### 3.2. Evaluation of the Effect of In Vivo Ultrasound Imaging

The ultrasound frequency of in vivo ultrasound imaging is 5.0 MHz, gain 51, MI ≤0.10. After injection of SPION contrast agent through the tail vein of the rat, the results showed that the carotid artery was imaged intact, the outline was clear, the contrast enhancement was uniform, and the carotid artery plaque was clear (see Figure 3).

### 3.3. Contrast-Enhanced Ultrasound Examination of the Expression of Inflammatory Adhesion Molecule VCAM-1 in Carotid Arteries

Theoretically, the VCAM-1 targeting contrast agent has a specific affinity for inflammation within the plaque and can effectively adhere to and reside in the inflammatory tissue. Contrast agents without VCAM-1 have no specific affinity for inflammation. Therefore, we observed the signal intensity of SPIONs carrying VCAM-1 antibody to model rats. The results show that the model A group has higher peak gray-scale video intensity and longer duration than the other two groups (see Figure 4). It shows that SPION contrast media carrying VCAM-1 antibody can be used to assess the inflammatory response of atherosclerotic lesions.

### 3.4. Serum Lipid Levels in Rats

By checking the levels of serum TC and LDL-C in rats, the results showed that the levels of TC and LDL-C in the model group were significantly higher than those in the control group (*P* < 0.05, see Figure 5). It shows that the cholesterol in the model group is at a high level, which accelerates the formation and development of plaque.

### 3.5. Pathological Examination of Rats

The HE staining observation revealed that the carotid arteries of the control group were clear. The thickness of smooth muscle is normal and uniform. No atherosclerotic plaque appeared (Figure 6(a)). In the carotid arteries of rats in the model group, obvious atherosclerotic plaques protruded into the lumen, which became smaller (Figure 6(b)).

### 3.6. Discussion

In order to study the ultrasound imaging effect of SPIONs, the effect of extracorporeal ultrasound imaging was first evaluated. We use latex tubes to simulate blood vessels and inject degassed water and SPION contrast media, respectively, to observe the imaging effects of SPIONs. The results showed that when degassed water was injected into the latex tube, only echo was seen on the wall of the tube and there was no echo in the lumen. When the SPION contrast agent is injected, there are obvious punctate strong echoes in the latex lumen, and the concentration of SPION contrast agent increases, and the echoes tend to be enhanced. In order to observe the imaging effect of SPION contrast agent in the carotid artery in rats, we used ApoE knockout rats to simulate the pathological model of human carotid inflammatory plaque [12]. Carotid atherosclerosis is a major risk factor for ischemic cardiovascular disease (CVD). ApoE is one of the most studied proteins in relationship to CVD and is crucial to the structural integrity of lipoproteins, plays a significant role in lipid metabolism, and is responsible for altering circulating levels of cholesterol. The APOE gene, located at chromosome 19q13.2, is polymorphic, and the three most common protein isoforms are E2, E3, and E4. Generally, the *ε*2 allele corresponds with lower mean plasma cholesterol levels and the *ε*4 allele with higher levels. ApoE polymorphisms do not appear to be an important risk factor for development of carotid plaque, but previous literature has demonstrated a significant relationship between the carrier status of the *ε*4 allele and carotid intima-media thickness (cIMT) [12].

After the SPION contrast agent was injected through the tail vein, the carotid arteries of rats with carotid plaques were observed. The results showed that the carotid arteries were intact with clear contours and uniform contrast enhancement. It shows that the SPION contrast agent shows better contrast enhancement effect. SPIONs have the advantages of good biocompatibility, easy surface modification, etc. and have broad application prospects in clinical medicine. According to related literature reports, a variety of SPIONs have been approved for MRI [13], but there are few reports in ultrasound imaging. Therefore, in this study, we loaded SPIONs on the surface of the polymer microbubble membrane shell to construct the SPION microbubble contrast agent that can achieve ultrasound imaging effects. And it was found that as the concentration of SPION microbubble contrast agent increased, the development continued to increase.

At present, the commonly used biomarkers for atherosclerosis research mainly focus on markers related to inflammation, such as intercellular adhesion molecule (ICAM-1) and vascular endothelial cell adhesion molecule 1 (VCAM-1), and are related to collagen decomposition. The markers include MMP-1, MMP-2, MMP-3, MMP-7, MMP-8, and MMP-9 [14–16]. VCAM-1 binds to other adhesion molecules to regulate immune surveillance and inflammatory response [17–19]. The expression of VCAM-1 is induced by the cytokine tumor necrosis factor alpha and interleukin-1 beta, adipokine visfatin, the atherogenic amino acid homocysteine, and atherogenic hyperglycemia [20–23]. Therefore, in order to explore the recognition effect of SPIONs on carotid inflammatory plaques, we then coupled a VCAM-1 protein that specifically binds to the inflammatory adhesion molecule on the microbubbles wrapped in SPIONs to form an antibody that carries VCAM-1 SPIONs. And the microbubble ultrasound contrast agent carrying VCAM-1 antibody was applied to the study of carotid inflammatory plaque in rats. We observed the signal intensity of SPIONs carrying VCAM-1 antibody to arteritis plaques. The results showed that the SPION contrast agent carrying VCAM-1 antibody had higher peak gray-scale video intensity and longer duration than the other two groups of contrast agents that did not carry VCAM-1 antibody contrast agent. It proves that SPION contrast media carrying VCAM-1 antibody can be used to assess the inflammatory response of atherosclerotic lesions. Bala et al. [24] used VCAM-1 as a target, radiolabeled with Fluorine-18, and used positron emission tomography to observe the expression of VCAM-1 in atherosclerotic model mice. The results showed that the probe's ability to recognize the expression of VCAM-1 is consistent with the results of this paper. Another study indicated that VCAM-1 displayed significantly higher expression on high-risk (symptomatic) vs. low-risk (asymptomatic) carotid plaques. Ultrasound contrast agents bearing ligands for VCAM-1 can sustain high-shear attachment and may be useful for identifying patients in whom more aggressive treatment is warranted [25]. However, Schumacher et al. found similar or lower VCAM-1 expression in symptomatic plaques; however, their manuscript does not show VCAM-1staining for evaluation, they do not evaluate the full carotid plaque, and most importantly, they were evaluating total VCAM-1 expression as opposed to only endothelial expression [26].

In order to verify whether the blood lipid levels of the model rats are at high levels after 16 weeks of feeding, we checked the levels of TC and LDL-C in the rats. The results showed that the levels of TC and LDL-C in the model group were significantly higher than those in the control group, at a higher level, and could be used in the next experiment. In this experiment, in order to verify whether the ultrasound imaging results of rats with carotid inflammatory plaques are consistent with the actual results, we performed pathological examinations on the carotid arteries of the rats. The results of HE staining showed that atherosclerotic plaques protruding into the lumen of the carotid arteries of the rats in the model group were consistent with the results of ultrasound imaging. Limitation is that, by design, we included in vivo who were symptomatic from their carotid disease, and it might be not conclusive considering our study model was nor representative of the whole spectrum of disease severity, bringing into question the generalizability of our results. Patients with carotid disease should be explored in the subsequent researched.

## 4. Conclusion

We demonstrated that SPION microbubble contrast agents have good imaging effects both *in vivo and in vitro*. And we observed the signal intensity of SPIONs carrying VCAM-1 antibody to arteritis plaques. The results showed that the SPION contrast agent carrying VCAM-1 antibody had higher peak gray-scale video intensity than the other two groups of contrast agents not carrying VCAM-1 antibody. Our data collectively indicated that SPIONs have excellent imaging effects in ultrasound imaging, can evaluate the inflammatory response of arterial plaque lesions, and are of great significance for the study of carotid inflammatory plaque changes.

## Figures and Tables

**Figure 1:** SPION microbubble contrast agent. (a) Microbubble optical microscopy image. (b) Transmission electron microscopy image.

**Figure 2:** The effect of in vitro ultrasound imaging. (a) The effect of different concentrations of SPION contrast agent on longitudinal section ultrasound imaging of latex tube. (b) The correlation between different concentrations of SPION contrast agent and the intensity of ultrasound grayscale video.

**Figure 3:** The effect of in vivo ultrasound imaging.

**Figure 4:** The signal intensity of SPIONs carrying VCAM-1 antibody to rats in the model group. (a) The contrast agent of SPIONs carrying VCAM-1 antibody. (b) A contrast agent for SPIONs that does not carry VCAM-1 antibody.

**Figure 5:** Serum lipid levels in rats. (a) Total cholesterol (TC); (b) low-density lipoprotein cholesterol (LDL-C). ∗∗∗∗ means that a *P* < 0.05 was considered statistically significant.

**Figure 6:** HE staining of rat carotid artery. (a) Control group (×200); (b) model group (×200).

## Data Availability

All the raw data could be accessed by contacting the corresponding author if any qualified researcher needs them.
